The article "Metabolomics Analysis Reveals Alterations in Cochlear Metabolic Profiling in Mice with Noise-Induced Hearing Loss" was published in 2022. Journal: Biomed Res Int.

# Metabolomics Analysis Reveals Alterations in Cochlear Metabolic Profiling in Mice with Noise-Induced Hearing Loss

**DOI:** 10.1155/2022/9548316

**Published:** 2022-05-06

**Authors:** Long Miao, Juan Zhang, Lihong Yin, Yuepu Pu

**Affiliations:** Key Laboratory of Environmental Medicine Engineering, Ministry of Education, School of Public Health, Southeast University, Nanjing 210009, China

## Abstract

Noise-induced hearing loss (NIHL) has always been an important occupational hazard, but the exact etiopathogenesis underlying NIHL remains unclear. Herein, we aimed to find metabolic biomarkers involved in the development of NIHL based on a mouse model using a gas chromatography coupled with mass spectrometry (GC-MS) metabolomics technique. We showed that the auditory brainstem response (ABR) thresholds at the frequencies of 4, 8, 12, 16, 24, and 32 kHz were all significantly elevated in the noise-exposed mice. Noise could cause outer hair cell (OHC) loss in the base of the cochlea. A total of 17 differential metabolites and 9 metabolic pathways were significantly affected following noise exposure. Spermidine acting as an autophagy modulator was found to be 2.85-fold higher in the noise-exposed group than in the control group and involved in *β*-alanine metabolism and arginine and proline metabolism pathways. Additionally, we demonstrated that LC3B and Beclin1 were expressed in the spiral ganglion neurons (SGNs), and their mRNA levels were increased after noise. We showed that SOD activity was significantly decreased in the cochlea of noise-exposed mice. Further experiments suggested that SOD1 and SOD2 proteins in the SGNs were all decreased following noise exposure. The upregulation of spermidine may induce LC3B- and Beclin1-mediated autophagy in the cochlear hair cells (HCs) through *β*-alanine metabolism and arginine and proline metabolism and be involved in the NIHL. ROS-mediated oxidative damage may be a pivotal molecular mechanism of NIHL. Taken together, spermidine can be regarded as an important metabolic marker for the diagnosis of NIHL.

## 1. Introduction

Noise is kind of unnecessary sound that can interfere with people's normal living such as rest, study, and work. Besides, noise is widely distributed in the human living environment, including traffic noise, construction noise, and occupational noise in the workplace. Noise pollution has become a severe public health problem and seriously threatens human's health and well-being. Available evidence has shown that elevated noise is significantly related to various diseases, such as hypertension, diabetes, heart failure, myocardial infarction, and stroke [1–3]. Moreover, noise is also an important industrial harmful factor, always endangering the health of workers [4]. Long-term noise exposure is known to impair the auditory function of the inner ear and cause permanent threshold shift (PTS) and eventually noise-induced hearing loss (NIHL), the second most common sensorineural hearing loss [5]. In addition, NIHL causes a negative impact on the development of social economy and social interaction and reduces quality of human life. According to WHO, approximately 10% of the population worldwide is exposed to high-intensity noise environments and faced the risk of developing NIHL [6]. It is worth noting that a previous study has reported that NIHL was the top two chronic occupational-related disease in China and was one-sixth of the annual increase in occupational diseases [7].

The article "Metabolomics Analysis Reveals Alterations in Cochlear Metabolic Profiling in Mice with Noise-Induced Hearing Loss" was published in 2022. Journal: Biomed Res Int.

Numerous studies have been performed to explore the mechanism of NIHL. Recent study has found that NIHL is associated with oxidative stress-induced sensory hair cell (HC) impairment, mediated by excessive production of reactive oxygen species (ROS) [8]. Experimental studies have provided clear evidence that ROS was a key mechanism contributing to the inner ear damage caused by noise exposure or ototoxic drug therapy [9]. Yang et al. [10] revealed that inflammation may be a crucial molecular mechanism involved in noise-induced cochlear damage. Miller et al. [11] found that 8-iso-prostaglandin F2*α*, a marker of ROS, was significantly increased in the inner ear of guinea pig following noise exposure, resulting in the reductions of blood flow in the cochlea and ultimately NIHL. Although many studies regarding NIHL were performed, the exact pathogenesis of NIHL has not been entirely illustrated.

Metabolomics, an effective technique, could systematically analyze metabolites and clarify the unique characteristics of the metabolic profile of disease, which could be used as significant biomarkers [12]. Wang et al. [13] reported that the endogenous metabolic alterations could reveal the body's direct biological responses to various stressors, including disease, environmental exposure, and nutritional imbalances. Metabolomics was widely applied to the diagnosis of various human diseases, such as cardiovascular diseases, cancer, and rheumatoid arthritis, along with neurodegenerative diseases [14–16]. Metabolomics has become a powerful tool to identify a potential biomarker for diagnosis, clinical therapeutic targets, and high-risk individual screening [17].

In this current study, firstly, we constructed a mouse model of NIHL using C57BL/6 mice; then, cochlear tissue samples were collected. Gas chromatography coupled with mass spectrometry (GC-MS) untargeted metabolomics was used to characterize the cochlear metabolic spectrum alterations between noise-exposed mice and control mice and to identify potential differential metabolites and pathways involved in the pathogenesis of NIHL.

The article "Metabolomics Analysis Reveals Alterations in Cochlear Metabolic Profiling in Mice with Noise-Induced Hearing Loss" was published in 2022. Journal: Biomed Res Int.

## 2. Materials and Methods

### 2.1. Animals

The flow chart designed in this study is presented in Figure 1. All animal experiments were performed on male C57BL/6 mice aged 6-8-weeks and weighting 18-24 g. A total of 40 mice were included. The mice were bred under specific controlled conditions with a temperature of 23°C, relative humidity of 50%, and a 12 h light/dark cycle with free access to standard laboratory food and distilled water. This study was approved by the Animal Care and Use Committee of Zhongda Hospital, affiliated to Southeast University (Grant No. 2020ZDSYLL150-P01). The experimental procedures were in accordance with the National Institutes of Health Guidelines for the Care and Use of Laboratory Animals. Moreover, every effort was made to decrease the number of animals used and protect them from suffering.

### 2.2. Noise Exposure and NIHL Model Construction

Mice were randomly divided into a noise-exposed group and non-noise-exposed (control) group (*n* = 20, each). A previous study reported that 120 dB sound pressure level (SPL) white noise exposure for 2 h condition could lead to NIHL and cochlear sensory hair cell degradation in mice [18]. In this study, broadband white noise exposure at 120 dB SPL for 4 h was carried out to construct an NIHL mouse model. Noise was produced by white noise synthesized with a specific digital signal processor (Intelligent Hearing Systems, Miami, FL, USA) connected to the computer and customized noise filters (Intelligent Hearing Systems, Miami, FL, USA). Noise signal was amplified and transmitted through speakers (RadioShack Corp., Fort Worth, TX, USA) installed on the walls of the exposure room. Each mouse of the noise-exposed group was maintained in a designed metal mesh cage, which was placed in the center of the acoustic room. Noise exposure intensity was determined with a sound level meter (TES-1350A, Taiwan). The mice of the control group were placed in a quite chamber and did not receive any disposal.

### 2.3. Auditory Brainstem Response (ABR) Examination

ABR was carried out immediately after noise exposure to evaluate the auditory threshold levels of each mouse. Each mouse was anesthetized by intraperitoneal injection of pentobarbital. Subdermal needle electrodes were fixed separately at the vertex of the head, right mastoid, and left hind leg. ABR tone burst stimulus was produced by Tucker-Davis Technologies system III equipment (TDT, Gainesville, FL, USA) in a sound insulation room. Auditory thresholds were assessed at six frequencies of 4, 8, 12, 16, 24, and 32 kHz initially from the sound intensity of 90 dB SPL and decreasing at intervals of 5 dB, until the visually recognizable ABR waveform could no more be tested. The auditory threshold was defined as the lowest level of the stimulus that could produce a visually identified response [19].

The article "Metabolomics Analysis Reveals Alterations in Cochlear Metabolic Profiling in Mice with Noise-Induced Hearing Loss" was published in 2022. Journal: Biomed Res Int.

### 2.4. Cochlea Surface Preparations and HC Counting

Three days following the ABR measurement, three mice in each group were anesthetized and decapitated for further experiment. Temporal bones were removed and placed into ice-cold Hanks' balanced salt solution (HBSS, Sigma-Aldrich, Saint Louis, MO, USA). The cochleae were washed with 0.1 M PBS, perfused with 4% paraformaldehyde, and then incubated at 4°C overnight. The cochleae were blocked using a 10% goat serum at 4°C overnight and incubated with anti-myosin7a antibody (1 : 100; Abcam, MA, USA) at 4°C overnight, followed by incubation with phalloidin conjugated with Alexa Fluor 488 (Life Technologies, CA, USA) for 2 h at room temperature to stain the stereocilia. DAPI (Life Technologies, CA, USA) was used to stain the nuclei. Samples were visualized using a Zeiss microscope at 40x magnification (Carl Zeiss, Oberkochen, Germany). The numbers of cochlear outer hair cells (OHCs) and inner hair cells (IHCs) were further quantified with ImageJ software (National Institutes of Health, Bethesda, MD, USA).

### 2.5. Chemicals and Reagents

All chemicals and solvents used were of analytical or high-performance liquid chromatography (HPLC) grade. Methanol, n-hexane pyridine, methoxylamine hydrochloride, and BSTFA were purchased from CNW Technologies GmbH (Düsseldorf, Germany). Moreover, the analytical reagent chloroform was purchased from Titan Scientific (Shanghai, China). L-2-Chloro-phenylalanine and 10 kinds of fat acid methyl ester were, respectively, purchased from Hengchuang Biotechnology (Shanghai, China), Larodan (Solna, Sweden), Nu-Chek (Minnesota, USA), and DR (Germany). Besides, Ultrapure water was obtained using the Milli-Q purify system (Millipore, USA).

### 2.6. Cochlear Sample Preparation and GC/MS Metabonomic Analysis

Six mice each of the control group and noise-exposed group were used for metabolomics analysis. To ensure the concentration of the cochlear sample for GC/MS analysis, a total of four cochleae from two mice were combined into one independent sample. Finally, three samples in each group were used for metabolomics analysis. Extracted cochleae were then frozen and stored at -80°C until analysis [20].

A 30 mg cochlea tissue from each sample was added to 20 *μ*L of L-2-chloro-phenylalanine and 600 *μ*L of mixture consisting of methanol : water (4 : 1) and then ground at 60 Hz for 2 min. After grinding, 120 *μ*L of chloroform was added and vortexed for 2 min, followed by ice water bath ultrasonic extraction for 10 min and standing for 30 min at -20°C. The sample was then centrifuged at 13000 rpm for 10 min at 4°C. After centrifugation, 200 *μ*L of the supernatant was collected and transferred to GC-MS vials followed by speed vacuum concentration using a centrifugal concentrator dryer. Further, 80 *μ*L methoxamine hydrochloride pyridine solution (15 mg/mL) was added and vortexed for 2 min and then incubated at 37°C for 90 min for oximation reaction. Subsequently, 50 *μ*L of BSTFA with 1% trimethyl-chlorosilane (TMCS) derivatization reagent, 20 *μ*L of n-hexane, and an alkane series (C8-C24) as the internal standard were mixed with the sample and then vortexed for 2 min followed by reaction at 70°C for 60 min. Finally, all samples were placed at room temperature for 30 min for GC-MS metabolomics analysis.

The article "Metabolomics Analysis Reveals Alterations in Cochlear Metabolic Profiling in Mice with Noise-Induced Hearing Loss" was published in 2022. Journal: Biomed Res Int.

Metabolomics analysis was performed with the Trace 1310/TSQ 9000 (Thermo Fisher Scientific, Waltham, MA, USA) system by a DB-5MS capillary column (30 m × 0.25 mm × 0.25 *μ*m, Agilent J&W Scientific, Folsom, CA, USA). The temperature of the inlet was set to 300°C, and the helium gas (>99.999%) was used as the carrier gas at a flow rate of 1.2 mL/min. The injection volume was 1 *μ*L. The initial temperature of the column was maintained at 60°C for 0.5 min, then increased to 125°C at 8°C/min, increased to 210°C at 5°C/min, increased to 270°C at 10°C/min, then increased to 305°C at 20°C/min, and kept at 305°C for 5 min. Moreover, the temperatures of the ion source and transmission line were 330°C and 280°C, respectively. The scanning mode was full scan, and mass scan range was 50-500 m/z. The metabolomics analysis was carried out by OE Biotech (Shanghai, China).

### 2.7. Multivariate Data Analysis and Metabolic Pathway Analysis

The raw data were firstly converted into abf format by the Analysis Base File Converter software and imported into MS-DIAL software for peak detection, identification, alignment, and filtering. The resulting data were exported and were analyzed using the untarget database of GC-MS from Lumingbio and NIST database. Unsupervised principal component analysis (PCA) was performed to evaluate the sample distribution, detect the outliers, and evaluate the data stability of the metabolomics analysis process. Supervised orthogonal partial least square-discriminant analysis (OPLS-DA) was conducted to distinguish the differences of metabolic profiles and find differential metabolites between noise-exposed and control groups. Multivariate data analysis was performed using SIMCA-P 14.1 software (Umetrics, Umeå, Sweden). Variable importance in projection (VIP), the weighted sum of the squares of the OPLS-DA analysis, could effectively indicate the importance of a variable to the model. Thus, in this study, the variables with the value of VIP > 1 were considered responsible for separation and defined as discriminative metabolites. The differential metabolite with a VIP > 1 and *P* < 0.05 was regarded as the potential biomarker responsible for NIHL. A visual heat map of the identified differential metabolites was produced using Multiple Experiment Viewer software.

The article "Metabolomics Analysis Reveals Alterations in Cochlear Metabolic Profiling in Mice with Noise-Induced Hearing Loss" was published in 2022. Journal: Biomed Res Int.

To investigate the metabolic pathways associated with noise exposure, differential metabolites were analyzed using MetaboAnalyst (http://www.metaboanalyst.ca). In detail, metabolic pathways were analyzed based on the differential metabolites identified by GC/MS metabolomics analysis. Metabolomics pathway analysis (MetPA) could identify significantly changed pathways under given experimental conditions. Pathway plots were performed based on the Kyoto Encyclopedia of Genes and Genomes (KEGG) database. KEGG pathway enrichment analysis of differentially metabolites was performed with hypergeometric distribution.

### 2.8. RNA Extraction, qRT-PCR, and Oxidative Stress Level Assay

Five mice each of control and noise-exposed groups were used. One cochlea of the same mouse was used for RNA extraction and qRT-PCR analysis, and the other cochlea was used for oxidative stress marker level detection. The total RNA was extracted by the TRIzol reagent (Invitrogen, Carlsbad, CA, USA). Reverse transcription was conducted with the Takara Prime Script RT reagent kit (Takara Bio, Clontech, Japan) according to the manufacturer's instructions. Specific primers designed from Generay Biotech (Shanghai, China) were applied to conduct qRT-PCR with the SYBR Green real-time PCR kits (Toyobo, Osaka, Japan). The primers were as follows: LC3BF: 5′-TTATAGAGCGATACAAGGGGGAG-3′ and LC3BR: 5′-CGCCGTCTGATTATCTTGATGAG-3′; Beclin1F: 5′-ATGGAGGGGTCTAAGGCGTC-3′ and Beclin1R: 5′-TGGGCTGTGGTAAGTAATGGA-3′; and *β*-actinF: 5′-GGGAAATCGTGCGTGAC-3′ and *β*-actinR: 5′-AGGCTGGAAAAGAGCCT-3′. The expression levels of LC3B and Beclin1 were normalized to the expression of *β*-actin. The results were calculated using the 2^−ΔΔCt^ method.

Evidence from related studies revealed that reactive oxygen species (ROS) was associated with autophagy and could trigger the cell defense autophagy pathway [21]. In addition, ROS was considered to play an essential role in the occurrence and development of inner ear injury induced by noise or ototoxic drug [22]. Superoxide dismutase (SOD) as the most important marker for the assessment of oxidative damage was measured to reflect the oxidative level. The activity of SOD in the cochlea was detected using the commercial chemical colorimetrical kits (Jiancheng Bioengineering, China) according to the manufacturer's instructions.

The article "Metabolomics Analysis Reveals Alterations in Cochlear Metabolic Profiling in Mice with Noise-Induced Hearing Loss" was published in 2022. Journal: Biomed Res Int.

### 2.9. Protein Extraction and Western Blotting

Cochlear tissues were homogenized in ice-cold RIPA lysis buffer together with phosphatase- and protease-inhibitors (Thermo Fisher Scientific, Waltham, MA, USA). Protein concentration was measured using a BCA assay kit (Beyotime Biotechnology, Shanghai, China). Equal amounts of cochlear proteins were separated using 12.5% SDS-PAGE and then transferred to PVDF membranes. The membranes were blocked using 5% nonfat milk in a TBST buffer at room temperature for 2 h and incubated with anti-SOD1 (1 : 1000, A12537, ABclonal Technology), anti-SOD2 (1 : 1000, A19576, ABclonal Technology), and GAPDH (1 : 1000, A19056, ABclonal Technology) overnight at 4°C. After, membranes were incubated using a HRP goat anti-rabbit IgG antibody (1 : 5000, AS014, ABclonal Technology) for 2 h at room temperature. Protein bands were captured using the Tanon-5200 Chemiluminescent Imaging System (Tanon Science & Technology, Shanghai, China). Three mice of each group were used for Western blotting, and three independent experiments of each target protein were performed.

### 2.10. Immunofluorescence

The cochleae were dissected and fixed in 4% paraformaldehyde buffered PBS for 24 h and decalcified using 10% EDTA. After decalcification, the cochleae were dehydrated overnight in 20% and 30% sucrose and then embedded in the optimal cutting temperature (OCT) glue (Sakura, USA). The cochleae were sectioned into 10 *μ*m thickness sections on a cryostat (Leica, Wetzlar, Germany). After, the sections were incubated with primary antibodies against LC3B (1 : 200, ABclonal Technology), Beclin1 (1 : 200, ABclonal Technology), SOD1 (1 : 200, ABclonal Technology), and SOD2 (1 : 200, ABclonal Technology) overnight at 4°C. Thereafter, the sections were incubated with a donkey anti-mouse IgG (H+L) conjugated with Alexa Fluor 488 (Life Technologies, CA, USA) and/or Alexa Fluor 555 donkey anti-rabbit IgG (H+L) (Life Technologies, CA, USA) at the room temperature for 2 h, followed by staining with DAPI (Life Technologies, CA, USA). Thereafter, the sections were rinsed and mounted with glycerin. The immunolabeling images were examined under a fluorescence microscope (Carl Zeiss, Oberkochen, Germany). Three mice of each group were used.

### 2.11. Statistical Analysis

The continuous variables were expressed as mean ± SD. Independent two-sample Student's *t*-test was carried out to determine the significant differences of data between two groups. Statistical analysis was performed with the SPSS 23.0 software (SPSS, Chicago, IL, USA). The statistical significance criterion was set with *P* value < 0.05. *P* value was indicated by asterisks (^∗^*P* < 0.05, ^∗∗^*P* < 0.01, and ^∗∗∗^*P* < 0.001).

The article "Metabolomics Analysis Reveals Alterations in Cochlear Metabolic Profiling in Mice with Noise-Induced Hearing Loss" was published in 2022. Journal: Biomed Res Int.

## 3. Results

### 3.1. ABR Threshold Analysis

The ABR thresholds of C57BL/6 mice between the noise-exposed group and control group are shown in Figure 2(a). There were significant differences in ABR thresholds at six frequencies between the two groups (*P* < 0.001). The ABR mean thresholds of noise-exposed mice were 83.50 ± 4.32 dB at 4 kHz, 79.50 ± 4.84 dB at 8 kHz, 73.75 ± 7.23 dB at 12 kHz, 73.75 ± 9.16 dB at 16 kHz, 81.25 ± 8.41 dB at 24 kHz, and 88.50 ± 2.86 dB at 32 kHz which were significantly greater than those of the control mice (47.50 ± 6.18 dB at 4 kHz, 34.25 ± 7.48 dB at 8 kHz, 28.25 ± 6.34 dB at 12 kHz, 30.00 ± 4.87 dB at 16 kHz, 37.50 ± 5.50 dB at 24 kHz, and 51.25 ± 3.93 dB at 32 kHz), suggesting that mice exposed to 120 dB for 4 h could develop NIHL.

### 3.2. Immunofluorescence Staining and HC Counting

To determine the pattern of HCs in the noise-exposed mice and control mice, immunofluorescence staining and HC counting experiments were performed. Immunofluorescence staining indicated that myosin7a- and phalloidin-positive OHC loss was significantly increased in the basal segment of the cochlea of noise-exposed mice compared to the control mice (Figures 2(b) and 2(c), *P* < 0.01, *n* = 3, each). The results suggested that the noise exposure condition of 120 dB SPL 4 h could result in NIHL and OHC degeneration and indicated that the NIHL model was successfully constructed in C57BL/6 mice.

### 3.3. Cochlear Metabolomics Profiles of the Noise-Exposed Mice and Control Mice

Unsupervised PCA was carried out to demonstrate the general overview of the clustering between groups. As shown in Figure 3(a), the scores plot of PCA suggested that the noise-exposed group was obviously separated from the control group along the PC1 and PC2, which explained 53.3% and 16.4% of the variation, respectively. Supervised clustering OPLS-DA has a higher discrimination ability and thus was implemented to describe the similarities and differences of samples between two groups. OPLS-DA indicated that there was distinct difference in score plots between the noise-exposed and control groups, suggesting that noise exposure caused significant metabolite profile alterations between the two groups (Figure 3(b)).

### 3.4. Identification of Cochlear Differential Metabolites

A total of 340 metabolites were identified based on GC/MS metabolomics analysis, but based on the OPLS-DA model analysis, 97 metabolites with VIP values > 1 were selected as discriminative metabolites and further verified by Student's *t*-test (*P* < 0.05). Finally, 17 differentially expressed metabolites were identified as displayed in Table 1. Among the 17 significantly changed metabolites, spermidine, 3-hydroxybutyric acid, and orotic acid were significantly upregulated in the noise-exposed group, compared to the control group. On the contrary, other 14 differential metabolites indicated downregulation. Interestingly, the spermidine, a crucial autophagy inducer, showed the most significant difference (*P* < 0.001), and its expression level increased up to 2.85-fold in the noise-exposed group compared to the control group. Moreover, to clearly display the differential metabolites between two groups, a visual clustering heat map based on the expressed levels of metabolites was produced and is displayed in Figure 4(a).

The article "Metabolomics Analysis Reveals Alterations in Cochlear Metabolic Profiling in Mice with Noise-Induced Hearing Loss" was published in 2022. Journal: Biomed Res Int.

### 3.5. Metabolic Pathway Analysis

The identified 17 significantly changed metabolites were selected for metabolic pathway enrichment analysis. Consequently, a total of nine metabolic pathways were significantly affected by noise exposure (*P* < 0.05), and the detailed analysis results are exhibited in Figure 4(b). All the nine apparently changed metabolic pathways including *β*-alanine metabolism, pyrimidine metabolism, cAMP signaling pathway, butanoate metabolism, synthesis and degradation of ketone bodies, arginine and proline metabolism, GABAergic synapse, and insulin secretion and purine metabolism. In addition, the enrichment degree of nine metabolic pathways was expressed by the rich factor, which was 0.09, 0.05, 0.08, 0.05, 0.17, 0.03, 0.11, 0.08, and 0.02, respectively (Table 2).

### 3.6. Autophagy Is Involved in NIHL Development via *β*-Alanine Metabolism and Arginine and Proline Metabolism

Among the nine significant metabolic pathways, we found that *β*-alanine metabolism was the most significant pathway (−log10(*P*) = 3.74). The significantly changed metabolites in the *β*-alanine metabolism pathway and the corresponding regulation genes are displayed in Figure 5(a). Spermidine, the significantly changed metabolite, was a critical compound involved in *β*-alanine metabolism and arginine and proline metabolism pathways. In this study, the level of spermidine was significantly increased in the noise exposure group compared with the control group (*P* < 0.001). As shown in Figure 5(a), SMS enzyme can convert spermine to spermidine, which can be converted into spermine by SMOX synthase. Spermidine could be synthesized into 4-aminobutanal by SPDH synthase. Then, ALDH2 synthase enzyme can utilize 4-aminobutanal as a substrate to synthesize 4-aminobutyric acid, a significantly downregulated metabolite in the noise exposure group. Furthermore, spermidine could be synthesized into *β*-aminopropion aldehyde under the action of the PAO4 synthase enzyme. Subsequently, ALDH3 synthetases synthesize *β*-alanine with *β*-aminopropion aldehyde. Previous studies confirmed that spermidine could trigger the autophagy process [23, 24]. Considering the close association between spermidine and autophagy, we further investigated whether changes in spermidine affect autophagy. Hence, the mRNA expression levels of LC3B and Beclin1, the main autophagy markers, were then explored. The results revealed that the mRNA levels of LC3B and Beclin1 were significantly increased in the cochleae from noise-exposed mice compared to those of the control group (Figure 5(b)) (*P* < 0.01). Moreover, we performed the immunofluorescence assay to explore the specific localization of LC3B and Beclin1 in the mouse cochlea. We found that LC3B and Beclin1 were expressed in the cochlear spiral ganglion neurons (SGNs) (Figures 5(c) and 5(d)).

The article "Metabolomics Analysis Reveals Alterations in Cochlear Metabolic Profiling in Mice with Noise-Induced Hearing Loss" was published in 2022. Journal: Biomed Res Int.

### 3.7. Measurement of Oxidative Damage

Oxidative stress is a significant mechanism involved in the inner ear injury caused by noise exposure. We measured the SOD level to determine the oxidative damage in the cochlea of mice from the two groups. The results showed that the activity of SOD in the cochlea was significantly decreased in the noise-exposed mice compared to the controls (Figure 6(a)). Western blot analysis revealed that SOD1 protein expression was significantly decreased in noise-exposed mice (Figures 6(b) and 6(c)). Similar expression was also observed in SOD2 protein (Figures 6(d) and 6(e)). Immunostaining indicated that SOD1 and SOD2 were expressed in SGNs. Weak staining of SOD1 and SOD2 was shown in SGNs of noise-exposed mice compared with the control mice (Figures 6(f) and 6(g)).

## 4. Discussion

NIHL has now become an urgent occupational health issue in the world, and its specific mechanism has not been elucidated. Hence, it is urgent to identify novel biomarkers and provide some scientific clues for understanding the mechanisms of NIHL. Metabolomics has been used to characterize the end products of metabolism and indicate the internal consequences of organisms to environmental factors and health effect. In this study, we aimed to explore the metabolic signature alterations in the cochlea and identify potential metabolic biomarkers and pathways involved in NIHL based on a NIHL mouse model by using a GC-MS platform.

First, a NIHL mouse model was established using male C57BL/6 mice exposed to 120 dB SPL for 4 h. Significantly higher ABR thresholds at 4, 8, 12, 16, 24, and 32 kHz and severe OHC loss in the basal part of the cochlea in the noise-exposed mice were observed, compared with the controls, indicating that the noise-exposed mice developed severe NIHL, and the NIHL mouse model was successfully constructed. These findings were consistent with previous studies suggesting that high-intensity noise could contribute to permanent NIHL coupled with OHC loss [18]. Importantly, the successful construction of the NIHL mouse model provides a strong basis for further metabonomic analysis. The metabonomic study showed that a total of 17 differentially metabolites were identified between two groups. Spermidine, 3-hydroxybutyric acid, and orotic acid showed a significantly high metabolic activity after noise exposure. In contrast, the expression of the other 14 metabolites could be significantly decreased after noise stimulation. The results also indicated that nine metabolic pathways were affected. These findings from current metabonomic study on the mouse cochlea provide strong evidence that high-level noise exposure could dramatically cause cochlear metabolic profiling alterations.

The article "Metabolomics Analysis Reveals Alterations in Cochlear Metabolic Profiling in Mice with Noise-Induced Hearing Loss" was published in 2022. Journal: Biomed Res Int.

Interestingly, among the metabolites, the spermidine, a crucial autophagy inducer, showed the most significant difference, and its expression level increased up to 2.85-fold in the noise-exposed group compared to the control group. Spermidine has been shown to have an important effect on reducing the risk of cardiovascular disease [25]. A recent animal study found that spermidine has an obvious protective effect against chemical-induced liver cancer and fibrosis and increased life expectancy by 25% [26]. Spermidine was also significantly associated with anti-inflammatory responses [27]. In addition, pathway enrichment analysis showed that spermidine is a major metabolite participating in both *β*-alanine metabolism and arginine and proline metabolism pathways, which were the most significant metabolic pathways affected by noise exposure. *β*-Alanine is a nonessential amino acid and key rate-limiting factor of carnosine participating in the process of carnosine synthesis. Previous studies have reported that carnosine is a crucial potent antioxidant and protects against oxidative stress [28]. Hence, *β*-alanine metabolism may have a close association with the generation of ROS in the cochlea, especially balancing the state between oxidation and antioxidant defenses. Oxidative stress has been confirmed to play a key role in noise exposure and ototoxic drug treatment-mediated inner ear injury [22, 29]. Furthermore, recent investigations have revealed that *β*-alanine may play an important role in changing stress metabolic response and participating in disease progression [30, 31]. In addition, a recent animal experimental study performed by He et al. [32] found that metabolic pathways including arginine and proline metabolism and purine metabolism were markedly altered by acoustic trauma. Given the special functional role of spermidine in the autophagy process, close relationship between *β*-alanine metabolism and ROS, and aberrantly changed arginine and proline metabolism induced by noise, we hypothesize that spermidine may be an important mediator of various pathophysiological factors of cochlear damage induced by noise stimulation, and the upregulation of spermidine may be involved in the pathological mechanism of cochlear injury in NIHL through regulating autophagy via *β*-alanine metabolism and arginine and proline metabolism pathways.

The article "Metabolomics Analysis Reveals Alterations in Cochlear Metabolic Profiling in Mice with Noise-Induced Hearing Loss" was published in 2022. Journal: Biomed Res Int.

Autophagy is defined as a primary biological process that maintains intracellular homeostasis through degrading damaged cellular components and proteins [33]. Previously, we performed metabolomics analysis of plasma samples from patients with NIHL and normal-hearing controls and found that autophagy emerged as a crucial role that may be involved in NIHL progression [21]. In this current study, spermidine, as a major metabolite involved in *β*-alanine metabolism and arginine and proline metabolism pathways, was observed to be significantly increased in noise-exposed mice. Previous studies confirmed that spermidine could trigger autophagy [23, 24]. Nowadays, increasing evidence indicates that autophagy is implicated in a great number of crucial physiological processes and involved in extensive diseases, including inflammation, cancer, neurodegenerative diseases, and cardiovascular diseases [34]. LC3B and Beclin1, core genes related to autophagy, were widely used as the markers to display autophagy. Therefore, we investigated the effects of noise on autophagy by determining the expression levels of LC3B and Beclin1 genes between two groups. The results showed that mRNA expression of LC3B and Beclin1 was elevated in the cochlea of noise-exposed mice, revealing that the autophagy process in the mouse cochlea could be significantly triggered by noise overstimulation via increasing the generation of spermidine and upregulation of autophagy gene expression. Consistently, recent studies also demonstrated that noise could promote the expression of LC3B and Beclin1 in the mouse cochlea and induce autophagy [9, 35]. Recent review revealed that autophagy has an essential function role in promoting auditory cell development and regulating functional maturation of the auditory system [36]. Besides, a previous study also showed that the deficiency of ATG5 leads to the degeneration of HCs and severe congenital hearing loss, indicating that autophagy plays a cytoprotective function in the cochlea [37]. We performed immunofluorescence experiments to know the specific localization of LC3B and Beclin1 proteins in the mouse cochlea. The data showed that both LC3B and Beclin1 were significantly expressed in the cochlear SGNs after noise exposure. The current results were like the previous findings indicating that LC3B and Beclin1 have positive expression in SGNs by noise stimulation or ototoxic drug exposure [9, 38]. SGNs have been shown to be more susceptible to various external stimuli, such as noise, ototoxic drugs, and inflammation stress [39]. Most hearing loss is caused by the failure and impairment of HCs and SGNs [40]. Our current findings suggest that spermidine, LC3B, and Beclin1 in the cochlea may act as important regulators involved in the development of NIHL response to noise stimulation. However, the roles of spermidine and autophagy mechanisms underlying NIHL remain unclear and needed to be functionally studied.

The article "Metabolomics Analysis Reveals Alterations in Cochlear Metabolic Profiling in Mice with Noise-Induced Hearing Loss" was published in 2022. Journal: Biomed Res Int.

Recent findings indicated that oxidative stress is a significant contributing factor involved in NIHL by damaging the cochlear HCs [8]. Previous research also revealed that ROS generation was a pathological phenomenon response to noise stimulation and appeared to be an active process in the cochlea [41]. Many antioxidants were found to be effective in protecting cochlear sensory HCs from the oxygen free radical damage [42]. In this study, we observed that the activity of SOD was decreased in the cochlea of noise-exposed mice, suggesting that SOD may be excessively consumed to remove the overproduction of oxygen free radicals and maintain the oxidative balance inside the cochlea. Similar results were also observed in the SOD1 and SOD2 protein levels showing that the expression levels were significantly decreased during noise exposure. These findings demonstrated that the decrease of SOD expression may be involved in the occurrence and development of NIHL. In addition, the results were consistent with the findings observed in the animal models, showing that SOD has a close association with ROS formation and might have an important role in protecting hearing function [43]. SOD has a protective effect on the cochlea against noise exposure. In contrast, SOD deficiency could increase the risk and susceptibility of NIHL [44]. A previous animal study showed a significant decrease in SOD expression in the cochlea of rats exposed to noise and showed that the higher the noise intensity, the lower the SOD expression level, which was consistent with our findings [45]. In conclusion, our findings suggest that ROS-mediated oxidative damage is an underlying pathological molecular mechanism of NIHL.

The article "Metabolomics Analysis Reveals Alterations in Cochlear Metabolic Profiling in Mice with Noise-Induced Hearing Loss" was published in 2022. Journal: Biomed Res Int.

This study was aimed at finding valuable metabolic biomarkers and pathways participating in NIHL by GC-MS metabolomics based on the NIHL mouse model and providing a novel scientific basis for further studies on the pathogenesis of NIHL, but potential limitations should be worthily considered. The number of samples eventually used for metabolomics analysis was relatively small because we made every effort to reduce the number of animals used and protect them from suffering. The current study was a pilot study aimed at identifying potential metabolites involved in the development of NIHL based on a model of NIHL using GC-MS metabolomics analysis. According to the results, totally, 17 differentially expressed metabolites were found to be closely associated with NIHL. Most importantly, it was the first study reporting that spermidine may induce LC3B- and Beclin1-mediated autophagy in the cochlear HCs through *β*-alanine metabolism and arginine and proline metabolism and be involved in the NIHL. However, as a pilot study, we did not perform experiments to examine the expression of these metabolites in HCs. In the following studies, we will carry out functional studies to explore the real expression of identified metabolites in HCs and to investigate their exact function role in the NIHL. In addition, we will study the spermidine-mediated autophagy mechanism underlying NIHL in vivo and in vitro.

## 5. Conclusions

In summary, our current study reveals that multiple metabolites and metabolic pathways were significantly altered by noise exposure. Our data provide the first evidence that spermidine may be an important regulator in the mouse cochlea triggered by noise stimulation, and the upregulation of spermidine might participate in the pathomechanism of cochlear HC damage in NIHL via inducing LC3B- and Beclin1-mediated autophagy activity by *β*-alanine metabolism and arginine and proline metabolism. Secondly, we demonstrate that ROS-mediated oxidative damage may be an underlying pathological molecular mechanism of NIHL. Therefore, spermidine can be regarded as an important metabolic marker for the diagnosis of NIHL. However, the exact role of spermidine and autophagy underlying NIHL remains unclear, and further studies are needed to illustrate this issue.

## Figures and Tables

**Figure 1:** The flow chart designed in this study.

**Figure 2:** A mouse model of NIHL was constructed using noise exposure condition of 120 dB SPL for 4 h. (a) Comparison of mean ABR hearing thresholds at the frequencies of 4, 8, 12, 16, 24, and 32 kHz between the noise-exposed and control mice (*n* = 20 each). (b) Myosin7a and phalloidin immunofluorescence staining of the mouse cochlea in two groups (*n* = 3 each). (c) Quantification of HCs in the apex, middle, and base segments of the cochlea in the two groups. Scale bars = 20 *μ*m. Data are represented as mean ± SEM. ^∗∗^*P* < 0.01 and ^∗∗∗^*P* < 0.001 compared to the control group.

The article "Metabolomics Analysis Reveals Alterations in Cochlear Metabolic Profiling in Mice with Noise-Induced Hearing Loss" was published in 2022. Journal: Biomed Res Int.

**Figure 3:** Cochlea metabolite profiles of noise-exposed mice are different from the control mice. (a) Scoring plots of the PCA model. (b) Scoring plots of the OPLS-DA model. Each point represents an independent sample; green dots represent samples in the noise-exposed group, and blue boxes represent samples in the control group.

**Figure 4:** Significantly altered metabolites and pathways caused by noise exposure. (a) A visual clustering heat map of the 17 differential metabolites (VIP > 1 and *P* < 0.05) between noise-exposed and control groups. (b) Scatter diagram of enriched KEGG pathways. Axis *x* represents the rich factor, and axis *y* represents the name of the enriched signaling pathway. The size of dots indicates the number of differential expression metabolites in a particular pathway, and the color of dots shows the range of *P* value.

**Figure 5:** Spermidine may participate in NIHL through activation of LC3B- and Beclin1-mediated autophagy via the *β*-alanine metabolism pathway and arginine and proline metabolism pathways. (a) Summary of the metabolites and corresponding regulation genes in the *β*-alanine metabolism pathway and arginine and proline metabolism pathways. (b) The relative mRNA expression of autophagy-related genes (LC3B and Beclin1). (c, d) Localization and expression levels of LC3B and Beclin1 proteins were detected by the immunofluorescence assay in the control group and noise group. The red and green fonts represent the up- and downregulation of differential metabolites in the solid line box; data are represented as mean ± SD. ^∗∗^*P* < 0.01 compared to the control group.

**Figure 6:** Detection of oxidative stress level in the cochlea after noise exposure. (a) Comparison of SOD activity in the cochlea between control and noise groups. (b, c) Western blotting showing the expression level of SOD1 protein in the mouse cochlea between the control and noise groups. (d, e) Western blotting showing the expression level of SOD2 protein in the mouse cochlea in the control and noise groups. (f, g) Localization and expression of SOD1 and SOD2 proteins were detected by the immunofluorescence assay in the control and noise groups. Data are represented as mean ± SD. ^∗^*P* < 0.05, ^∗∗^*P* < 0.01, and ^∗∗∗^*P* < 0.001 compared to the control group.

**Table 1:** Endogenous differential metabolites of the cochlea between noise-exposed and control groups.

No.	Metabolites	Retention time (min)	Quant mass (*m*/*z*)	VIP	*P* value	Fold change
1	Spermidine	14.89	100.02	2.31	<0.001	2.85
2	3-Hydroxybutyric acid	8.15	147.00	2.25	0.013	2.85
3	Glucose-6-phosphate	20.40	147.03	2.25	0.021	0.36
4	Phenylethylamine	9.99	299.46	2.23	0.045	0.33
5	Thymine	12.68	255.01	2.19	0.049	0.32
6	D-Fructose	16.44	102.97	2.12	0.047	0.35
7	3,4-Dihydroxycinnamic acid	20.39	219.10	2.03	0.011	0.42
8	Arbutin	14.84	243.08	1.96	0.036	0.42
9	Hypoxanthine	21.23	264.99	1.93	0.010	0.46
10	4-Aminobutyric acid	15.46	174.02	1.84	0.028	0.48
11	5,6-Dihydrouracil	14.84	128.01	1.77	0.031	0.50
12	Triacontanol	24.45	102.91	1.67	0.019	0.55
13	Orotic acid	20.07	254.00	1.66	0.009	1.78
14	1-Hexacosanol	24.44	299.17	1.64	0.020	0.56
15	Adenine	12.64	239.03	1.51	0.045	0.58
16	4-Aminobenzoicacid	12.50	103.03	1.26	0.050	0.68
17	Salicylaldehyde	11.99	192.98	1.26	0.033	0.70

VIP: variable importance in projection.

The article "Metabolomics Analysis Reveals Alterations in Cochlear Metabolic Profiling in Mice with Noise-Induced Hearing Loss" was published in 2022. Journal: Biomed Res Int.

**Table 2:** Significantly altered pathways affected by noise exposure.

No.	Pathway name	Total compounds^1^	Hits^2^	*P* value	−Log10(*P* value)	FDR correction^3^	Rich factor^4^
1	*β*-Alanine metabolism	32	3	<0.001	3.74	0.006	0.09
2	Pyrimidine metabolism	65	3	0.001	2.83	0.024	0.05
3	cAMP signaling pathway	25	2	0.004	2.44	0.038	0.08
4	Butanoate metabolism	42	2	0.010	2.00	0.080	0.05
5	Synthesis and degradation of ketone bodies	6	1	0.022	1.66	0.096	0.17
6	Arginine and proline metabolism	78	2	0.032	1.49	0.096	0.03
7	GABAergic synapse	9	1	0.033	1.48	0.096	0.11
8	Insulin secretion	12	1	0.044	1.36	0.106	0.08
9	Purine metabolism	95	2	0.046	1.33	0.106	0.02

^1^Total compounds: the total number of compounds in the pathway. ^2^Hits: the number of differential metabolites involved in this pathway. ^3^FDR correction: the *P* value adjusted by false discovery rate. ^4^Rich factor: the ratio of the number of differential metabolites to the total number of metabolites in this pathway.

## Data Availability

The data used to support the findings of this study are available from the corresponding author upon request.
